This article has been retracted.

# Long noncoding RNA ANRIL is activated by hypoxia-inducible factor-1α and promotes osteosarcoma cell invasion and suppresses cell apoptosis upon hypoxia

**DOI:** 10.1186/s12935-016-0349-7

**Published:** 2016-09-23

**Authors:** Xiaokang Wei, Chuanshun Wang, Chunhui Ma, Wei Sun, Haoqing Li, Zhendong Cai

**Affiliations:** Department of Orthopaedics, Shanghai General Hospital, Shanghai Jiao Tong University School of Medicine, No 100 Hanning Road, Shanghai, 200080 People’s Republic of China

**Keywords:** Osteosarcoma, Long noncoding RNA, Hypoxia, HIF-1α, ANRIL

## Abstract

**Background:**

Osteosarcoma is the most common malignancy of bone. Intratumoral hypoxia occurs in many solid tumors, where it is associated with the development of aggressive phenotype. ANRIL has been shown to be a long noncoding RNA that facilitates the progression of a number of malignancies. Yet, few studies have explored the expression pattern of ANRIL in osteosarcoma and the effect of hypoxia on ANRIL.

**Methods:**

We evaluated the expression levels of ANRIL in osteosarcoma tissues, adjacent normal tissues and cells with quantitative real-time polymerase chain reaction. Multiple approaches including luciferase reporter assay with nucleotide substitutions, chromatin immunoprecipitation assay and electrophoretic mobility shift assay were used to confirm the direct binding of HIF-1α to the ANRIL promoter region. SiRNA-based knockdown and other molecular biology techniques were employed to measure the effect of HIF-1α on the expression of ANRIL.

**Results:**

We found that the expression of ANRIL was upregulated in 15 pairs of osteosarcoma compared with adjacent normal tissues. We found that hypoxia is sufficient to upregulate ANRIL expression in osteosarcoma cells (MNNG and U2OS). HIF-1α directly binds to the putative hypoxia response element in the upstream region of ANRIL. What’s more, siRNA and small molecular inhibitors-mediated HIF-1α suppression attenuated ANRIL upregulation under hypoxic conditions. Upon hypoxia, ANRIL promoted cancer cell invasion and suppressed cell apoptosis.

**Conclusion:**

Taken together, these data suggest that HIF-1α may contribute to the upregulation of ANRIL in osteosarcoma under hypoxic conditions. ANRIL is involved in hypoxia-induced aggressive phenotype in osteosarcoma.

## Background

Osteosarcoma (OS) is a highly malignant tumor of bone that occurs mainly in the extremities of juvenile groups [1, 2]. The 5-year event-free survival rate (EFS) for patients diagnosed with localized disease has improved since the combined used of chemotherapy, radiotherapy and surgical ablation of the primary tumor. However, the 5-year survival rate of osteosarcoma patients with metastases is lower than 30 % [3, 4]. Accordingly, the leading cause of dismal outcomes in osteosarcoma is tumor metastasis. Thus, targeting osteosarcoma metastasis may be a promising strategy in the treatment of human osteosarcoma. However, little progress has been made in this area as the molecular mechanisms underlying osteosarcoma invasion and metastasis remain poorly understood.

Hypoxia have been shown to increase risks of invasion, metastasis, treatment failure, and patient mortality in the majority of solid tumors, including osteosarcoma [5, 6]. The hypoxia inducible factor-1 (HIF-1) complex plays a key role in mediating hypoxic response [7]. HIF-1 is a heterodimeric transcription factor formed by HIF-1α and HIF-1β [8]. Previous studies have showed that hypoxia-inducible factor-1 alpha (HIF-1α), a transcription factor that is stabilized under hypoxic conditions, regulates the expression of multiple target genes by binding to the Hypoxia Responsive Elements (HREs, 5′-RCGTG-3′) in their enhancers or promoters regions [9]. HIF-1α accumulation help cancer cells adapt to and survive in hypoxic conditions, leading to poor therapeutic responses, decreased overall survival and disease-free survival in osteosarcoma patients [10–12]. Thus, it is vital to identify hypoxia-responsive genes for the development of effective treatments.

In addition to regulating protein-coding genes, including but not limited to, vascular endothelial growth factor A (VEGFA), angiopoietin-like 4 (ANGPTL4), phosphoglycerate kinase 1 (PGK1), hexose kinase 2 (HK2) and carbonic anhydrase IX (CAIX) [12], hypoxia/HIF-1α has been revealed to regulate the expression of miRNAs [13, 14]. Long noncoding RNAs are an important a subclass of noncoding RNAs, which are longer than 200 nucletides (nts) in length and with little protein-coding potential. A growing volume of literature has confirmed the vital role that lncRNAs play in cancer biology [15–17]. However, the effect of hypoxia/HIF-1α on lncRNAs remains to be explored.

Long noncoding RNA ANRIL (CDKN2B antisense RNA 1) is transcribed as a 3.8-kb lncRNA in the opposite direction from the INK4B-ARF-INK4A gene cluster [18]. ANRIL has been demonstrated to exert oncogenic activity in a variety of carcinomas [19–21]. The expression pattern of ANRIL in osteosarcoma tissues and in osteosarcoma cells under hypoxic conditions remain to be elucidated.

In the present study, we would like to explore the expression pattern and function of ANRIL in hypoxic osteosarcoma cells. We found that HIF-1α transcriptionally activated ANRIL via directly binding to HREs in the upstream region of ANRIL upon hypoxia. The upregulation of ANRIL facilitated invasion of hypoxic osteosarcoma cells and inhibited cell apoptosis. Our data provides novel insights into the molecular mechanisms of how hypoxia/HIF-1α contributes to oncogenic phenotype of osteosarcoma and the involvement of ANRIL in the more aggressive cancer cell phenotype under hypoxic conditions.

## Methods

### Human osteosarcoma samples

A total of 15 osteosarcoma samples were collected postoperatively from patients who underwent surgical resection between 2006 and 2011 at the Department of Orthopedics, Shanghai Jiao Tong University Affiliated Sixth People’s Hospital (Shanghai, China). Informed consent was obtained from the patients enrolled in this study. The study was approved by the Ethics Committee of Shanghai Jiao Tong University (2015-DY-126).

### Cell culture

The MNNG and U2OS cell lines were purchased from the ATCC. The cell lines were grown in Dulbecco’s Modified Eagle Medium (DMEM, Gibco BRL, Grand Island, NY, USA) supplemented with 10 % fetal bovine serum (FBS, HyClone, Camarillo, CA, USA) as well as 100 U/ml penicillin and 100 μg/ml streptomycin (Invitrogen, Carlsbad, CA, USA). Cells were maintained in a humidified incubator at 37 °C in the presence of 5 % CO_2_. All cell lines have been passaged for fewer than 6 months. Hypoxia treatment (1 % O_2_, 5 % CO_2_, and 94 % N_2_) was performed in hypoxia Workstation (InVIVO2). The cells were incubated under hypoxic conditions for 24 h. HIF-1α specific inhibitor 3-(5′-hydroxymethyl-2′-furyl)-1-benzylindazole (YC-1) was purchased from Sigma (Sigma Aldrich, St. Louis, MO, USA) and resolved in dimethyl sulfozide (DMSO). YC-1 treatment was used at a final concentration of 40 μM. YC-1 and equal volume of control (DMSO) were added into the culture medium 12 h before hypoxia treatment.

### RNA extraction and quantitative real-time PCR

Total RNA was extracted from cancer cells utilizing the Trizol reagent (Invitrogen, Carlsbad, CA, USA) according to the manufacturer’s instructions and quantified with Nanodrop 2000 (Thermo Fisher Scientific, Waltham, MA, USA). First-strand cDNA was generated with the Primer-Script™ one step RT-PCR kit (TaKaRa, Dalian, China). Quantitative real-time polymerase chain reaction (qRT-PCR) was performed with SYBR Green premix Ex Taq (TaKaRa) with β-actin as an internal control. MRNA values were normalized to that of β-actin. The relative expression of mRNA was calculated with the 2^−ΔΔCt^ method. Each sample was repeated in triplicate. QRT-PCR data were analyzed and converted to relative fold changes. The primer sequences used in the present study were as the followings: ANRIL, 5′-TTGTGAAGCCCAAGTACTGC-3′(forward), 5′-TTCACTGTGGAGACGTTGGT-3′(reverse); HIF-1α, 5′-CATCTCCATCTCCTACCCACA-3′(forward), 5′-CTTTTCTGCTCTGTTTGGTG-3′(reverse); GAPDH, 5′-AGAAGGCTGGGGCTCATTTG-3′(forward), 5′-AGGGGCCATCCACAGTCTTC-3′(reverse); β-actin, 5′-CTGGGACGACATGGAGAAAA-3′(forward), 5′-AAGGAAGGCTGGAAGAGTGC-3′(reverse).

### Western blot analysis

Cell lysates were extracted from cultured cells with RIPA buffer (Cell Signaling Technology) supplemented with the protease inhibitors. The lysates were subjected to ultrasonication and centrifugation. The protein concentrations were determined with the BCA Protein Assay Kit (Pierce). Equal amounts (30–40 μg) of proteins samples were separated by 8–12 % SDS–polyacrylamide gel electrophoresis and then transferred onto a nitrocellulose filter membranes (Millipore). After blocking in phosphate-buffered saline/Tween-20 containing 5 % non-fat milk, the membrane was immunoprecipitated with indicated primary antibodies overnight at 4 °C: rabbit polyclonal anti-human HIF-1α antibody (1:1000, Abcam), rabbit polyclonal anti-human Bcl-2 antibody (1:500, Abcam), rabbit polyclonal anti-human Bax antibody (1:500, Abcam), and rabbit polyclonal anti-human β-actin antibody (1:1000, Abcam). The membranes were washed with TBST (3 × 5 min), and then immunoprecipitated with the secondary antibody [HRP-conjugated goat anti-rabbit IgG antibody (Abcam)] for 1 h at room temperature. Subsequent visualization was detected with SuperSignal West Femto Maximum Sensitivity Substrate (Thermo Fisher Scientific). Intensities of the bands were normalized to the corresponding β-actin bands.

### Plasmid construction

The ANRIL promoter constructs were generated using PCR-based amplification with human genomic DNA as the template and was subcloned in the pGL3 basic firefly luciferase reporter. The HRE mutations were created using a Quick-change Multi Site-Directed Mutagenesis Kit (Stratagene, La Jolla, CA, USA) with ANRIL promoter plasmid as the template. The primers for Site-directed mutagenesis were: 5′-CAAATATGAGAAATGTATCGAGCTCCATCTGGGTAAGAC-3′(forward), 5′-GTCTTACCCAGATGGAGCTCGATACATTTCTCATATTTG-3′(reverse).

### Cell transfection

ANRIL specific siRNA, HIF-1α siRNA and Allstars Negative Control siRNA were purchased from Biotend (Shanghai, China). HIF-1α siRNA, 5′-CCGCTGGAGACACAATCATAT-3′; ANRIL siRNA-1, 5′-GGUCAUCUCAUUGCUCUAU-3′; ANRIL siRNA-2, 5′-AAAUCCAGAACCCUCUGACAUUUGC-3′; siRNA control, 5′-UUCUCCGAACGUGUCACGUTT-3′. Vector were transfected into cells by Lipofectamine-mediated gene transfer according to the manufacturer’s protocol. For RNA extraction and western blotting assays, cells were used 48 h after transfection.

### Luciferase reporter assay

HIF-1α siRNA and the ANRIL promoter/luciferase reporter construct were cotransfected into osteosarcoma cells by Lipofectamine 2000-mediated gene transfer. Each sample was cotransfected with the pRL-TK plasmid in order to monitor transfection efficiency (Promega, Madison, WI, USA). Luciferase assays were carried out utilizing the dual-luciferase reporter assay system kit (Promega). The luciferase expression was measured with Modulus single-tube multimode reader (Promega). The relative luciferase activity was normalized to the renilla luciferase activity.

### Electrophoretic mobility shift assay (EMSA)

OSTEOSARCOMA cells were incubated under hypoxic conditions for 24 h. EMSA was carried out utilizing a light shift chemiluminescent EMSA kit (Pierce). Nuclear proteins from OSTEOSARCOMA cells were prepared using NE-PER nuclear and cytoplasmic extraction reagents (Pierce, Rockford, IL, USA). Nuclear proteins (4 μg) were incubated with binding buffer [2.5 % glycerol, 5 mM MgCl_2_, 0.05 % NP-40, 1 μg poly(dI–dC), 10 mM Tris, 50 mM KCl, 1 mM DTT, pH 7.5] with or without of 200-fold (3 pmol) unlabeled probes (cold probe or mutant probe) for 20 min, followed by the incubation with the biotin labeled probes (10 fmol) for 20 min. Samples were electrophoresed on a 6 % polyacrylamide gel. The probes used were as the followings: HRE probe, 5′-AATGTATCACACGCCATCTGGG-3′; HRE mutant probe, 5′-CGAGCGCAGTGGCATGGGGCTGTAATCCCA-3′.

### Chromatin immunoprecipitation (ChIP) assay

Chromatin immunoprecipitation (ChIP) assays were carried out using the EZ ChIP Chromatin Immunoprecipitation Kit (Millipore, Bedford, MA, USA) according to the manufacturer’s protocol. Briefly, Chromatin was sonicated on ice to an average length of 200–300 bp in an ultrasound bath. Human IgG was employed as the negative control. Chromatin was immunoprecipitated with rabbit polyclonal anti-human HIF-1α antibody (Abcam, Cambridge, MA, USA). ChIP-derived DNA was quantified using qRT-PCR. Quantitative PCR reactions were then performed on real-time PCR machine (Realplex2, Eppendorf) with ChIP primers: 5′-AAGATCTCGGAACGGCTCT-3′(forward), 5′-TCAGGTGACGGATGTAGCTA-3′(reverse).

### Cell viablity assay

Cell viability assays were performed utilizing the CCK-8 assay kits following by the manufacturer’s protocol. Cells transfected with desired vector were seeded into the 96-well plates at an initial density of 5000 cells/well and cultured under hypoxic conditions. At the indicated time points, CCK-8 solution 10 µl was added into each well and incubated for 2 h. The absorbance was determined by scanning at 450 nm with a microplate reader. Data were presented as the percentage of viable cells as the followings: relative viability (%) = (A450_treated_ − A450_blank_)/(A450_control_ − A450_blank_) × 100 %.

### Cell apoptosis assay

Cells transfected with desired vector were seeded into the 6-well plates and cultured under hypoxic conditions for 48 h. The cultures were then stained with annexin V-FITC and propidium iodide (Beyotime, Haimen, China) following the manufacture’s instructions and examined using a flow cytometer (Becton–Dickinson, USA).

### Cell invasion assay

Cells transfected with desired vector (2 × 10^5^ in 100 µl serum-free medium) were seeded in the upper chamber of an insert (8.0 µm, Millipore, MA). The insert was pre-coated with Matrigel (Sigma, USA). The lower chamber was added with 400 µl of culture medium supplemented with 10 % FBS for 24 h hypoxia treatment before final examination. The cells on the upper surface that didn’t invade were wiped off with a cotton swab, whereas cells on the lower membrane surface were fixed with methanol for 15 min and stained with 0.01 % crystal violet in PBS for 10 min. Cells from three random fields were counted under a phase contrast microscope (original magnification, ×200) and the relative number was determined. Experiments were repeated in triplicate.

### Statistical analysis

All statistical analyses were performed using SPSS 17.0 (SPSS, Chicago, USA). All data were presented as mean ± standard error from three independent experiments. Statistical evaluations were analyzed with independent student’s t test unless otherwise indicated. A two-sided *P* value less than 0.05 was considered to be statistically significant.

## Results

### Hypoxia transcriptionally activated ANRIL in osteosarcoma cells

To start with, we examined the expression pattern of ANRIL in osteosarcoma tissues. According to the results of qRT-PCR, the expression levels of ANRIL were significantly higher in osteosarcoma tissues compared with adjacent normal tissues (n = 15, P < 0.001; Fig. 1a). As ANRIL was frequently upregulated in osteosarcoma, we would like to determine the transcriptional factors that contributed to its upregulation. In the first place, we examined the effect of hypoxia on the expression level of ANRILA. Hypoxia obviously increased the transcript levels of ANRIL in MNNG and U2OS cells (Fig. 1b). Meanwhile, hypoxia markedly enhanced the promoter activities of ANRIL (Fig. 1c). Together, it suggests that hypoxia promoted the transcriptional activity and expression level of ANRIL in osteosarcoma cells.

**Fig. 1:** Hypoxia upregulates ANRIL expression in osteosarcoma cells. **a** Expression level of ANRIL by qRT-PCR in 15 osteosarcoma tissues and paired non-tumor tissues. GAPDH was used as a loading control. **b** ANRIL expression under both normoxic and hypoxic conditions were analyzed by real-time PCR. **c** ANRIL promoter activity under both normoxic and hypoxic conditions were analyzed by luciferase assay (**, *P* < 0.01, n = 3). β-actin was used as the internal control (**, *P* < 0.01, n = 3)

### HIF-1α directly binds to hypoxia responsive elements (HREs) of the ANRIL promoter region under hypoxic conditions

We sought to investigate whether HIF-1α took a part in upregulating the expression level of ANRIL under hypoxic conditions. We identified one putative binding site for HIF-1 (HRE, −714 to −705 bp) in the upstream region of ANRIL with online bioinformatical software programs MatInspector (http://www.genomatix.de/online_help/help_matinspector/matinspector_help.html) (Fig. 2a). We detected the expression of HIF-1α under normoxic and hypoxia conditions. Western blotting analysis demonstrated that hypoxia obviously upregulated the protein levels of HIF-1α, whereas hypoxia had no effects on the mRNA levels of HIF-1α (Fig. 2b, c). The direct interaction between HIF-1α and putative HRE was confirmed with the EMSA assay (Fig. 2d). Furthermore, HIF-1α immunoprecipitates were highly enriched in the DNA fragments compared with negative control IgG immunoprecipitates in the ChIP assay (Fig. 2e). Together, it suggests that HIF-1α directly binds to hypoxia responsive elements (HREs) of the ANRIL promoter region upon hypoxia in both MNNG and U2OS cells.

**Fig. 2:** HIF-1α binds to hypoxia responsive elements of the ANRIL promoter under hypoxic conditions. **a** Schematic representation of the putative binding sites of hypoxia responsive elements (HREs) in the ANRIL promoter. **b** HIF-1α mRNA levels under both normoxic and hypoxic conditions (24 h) were analyzed by real-time PCR. β-actin was used as the internal control. **c** HIF-1α protein levels under both normoxic and hypoxic conditions were analyzed by Western blotting. β-actin was used as the internal control (**, *P* < 0.01, n = 3). **d** EMSA showed the interaction of HIF-1α with the ANRIL promoter in vitro. **e** ChIP showed the interaction of HIF- 1α with the ANRIL promoter. The HIF-1α antibody effectively enriched the DNA sequence covering the putative binding element. Normal rabbit IgG was used as a negative control, and an anti-HIF-1α polymerase antibody was used as a positive control. Sonicated DNA fragments were used as input

### HIF-1α potently induces ANRIL expression in osteosarcoma cells upon hypoxia

To explore whether HIF-1α transcriptionally activates ANRIL expression in osteosarcoma cells under hypoxic conditions, we constructed the wild and mutant type of HRE in the promoter region of ANRIL. A significant reduction in the ANRIL promoter activity was observed when we mutated the putative HREs in both MNNG and U2OS cells upon hypoxia (Fig. 3a). A HIF-1α specific siRNA was transfected in MNNG and U2OS cells to suppress HIF-1α expression under hypoxic conditions. HIF-1α specific siRNA potently decreased the mRNA and protein levels of HIF-1α (Fig. 3b, c). Meanwhile, HIF-1α specific siRNA significantly reduced the promoter activities (Fig. 3d) and transcript levels (Fig. 3e) of ANRIL in both MNNG and U2OS cells. In the meantime, HIF-1α-specific inhibitor YC-1 significantly reduced the mRNA (Fig. 3f) and protein levels (Fig. 3g) of HIF-1α under hypoxic conditions. YC-1 also ameliorated the upregulation of ANRIL in hypoxic osteosarcoma cells (Fig. 3h). Collectively, these data showed that HIF-1α could transcriptionally activate ANRIL in hypoxic osteosarcoma cells.

**Fig. 3:** HIF-1α enhances ANRIL expression in osteosarcoma cells. **a** Osteosarcoma cells were transfected with HRE-mutant ANRIL promoter constructs. ANRIL promoter activity was detected by luciferase assay (**, *P* < 0.01, n = 3). **b** HIF-1α mRNA levels were analyzed by real-time PCR after siRNA knockdown of HIF-1α. β-actin was used as an internal control (**, *P* < 0.01, n = 3). **c** HIF-1α protein levels were analyzed by Western blotting after HIF-1α knockdown. β-actin was used as the internal control. (**, *P* < 0.01, n = 3). **d** Effect of HIF-1α silencing on ANRIL promoter activity was detected by luciferase assay (**, *P* < 0.01, n = 3). **e** Effect of HIF-1α silencing on ANRIL expression was detected by real-time PCR. β-actin was used as an internal control (**, *P* < 0.01, n = 3). **f** HIF-1α mRNA levels were analyzed by real-time PCR after treatment with YC-1 HIF-1α-specific inhibitor (40 μM). β-actin was used as an internal control (**, *P* < 0.01, n = 3). **g** HIF-1α protein levels were analyzed by Western blotting after treatment with YC-1 (40 μM). β-actin was used as the internal control (**, *P* < 0.01, n = 3). **h** Effect of YC- 1 on ANRIL expression was detected by real-time PCR. β-actin was used as an internal control (**, *P* < 0.01, n = 3)

### Effects of ANRIL silencing on viability and apoptosis of hypoxic osteosarcoma cells

To investigate the biological effects of ANRIL under hypoxic conditions, we transfected U2OS cells with the most efficient ANRIL specific siRNA that have been confirmed in other studies [19]. The hypoxia-induced ANRIL expression was knocked down by ANRIL specific siRNAs (Fig. 4a). ANRIL silencing reduced the hypoxic cell viability compared to the negative control cells (Fig. 4b). Furthermore, ANRIL silencing increased the apoptosis rate of U2OS cells compared to the negative control cells under hypoxic conditions (Fig. 4c). ANRIL-knocked down cells demonstrated increased Bax/Bcl-2 ratio under hypoxic conditions (Fig. 4d). Thus, it indicates that ANRIL increases cell viability and inhibits apoptosis of osteosarcoma cells under hypoxic conditions.

**Fig. 4:** Effects of ANRIL silencing on the viability and apoptosis of hypoxic osteosarcoma cells. **a** Knockdown efficiency of ANRIL siRNA was detected by real-time PCR. β-actin was used as the internal control (**, *P* < 0.01, n = 3). **b** Cell viability of ANRIL-silenced and negative control U2OS cells cultured under hypoxic conditions was detected by CCK-8 assay. Data are presented as a percentage of the control group (**, *P* < 0.01, n = 3). **c** Apoptosis of ANRIL-silenced U2OS cells and negative control cells under hypoxia conditions was measured by flow cytometry (**, *P* < 0.01, n = 3). **d** Bax and Bcl-2 protein levels were analyzed by Western blotting after ANRIL knockdown. β-actin was used as the internal control. (**, *P* < 0.01, n = 3). Data represent the mean ± S.D

### ANRIL silencing attenuated hypoxia-induced invasion in osteosarcoma cells

In the functional aspect, we investigated the effects of ANRIL on invasive capacity of osteosarcoma cells. Hypoxia significantly increased the invasive potencies of U2OS cells (Fig. 5a, b). However, such as effect was attenuate by ANRIL silencing (Fig. 5a, b). These data suggest that ANRIL is involved in hypoxia-mediated invasion of osteosarcoma cells.

**Fig. 5:** Effects of ANRIL silencing on the invasion of hypoxic osteosarcoma cells. **a**, **b** Invasion of U2OS cells can be enhanced by hypoxia conditions, and can be rescued by ANRIL silencing (**, *P* < 0.01, n = 3). Data represent the mean ± S.D

## Discussion

It has been well recognized that hypoxia results in the transformation of cancer cells into more aggressive phenotypes through the regulation of oncogenes that promote the progression and metastasis of cancer [5–7]. However, whether lncRNA is involved in such a process remains largely elusive. The present study characterized ANRIL as a hypoxia-inducible lncRNA that is important for the hypoxia-mediated aggressive phenotype.

Long noncoding RNA ANRIL (CDKN2B antisense RNA 1) is transcribed as a 3.8-kb lncRNA in the opposite direction from the INK4B-ARF-INK4A gene cluster [18]. ANRIL has been demonstrated to exert oncogenic activity in a variety of carcinomas [19, 20]. Yet, few studies have focused on the transcriptional factors that contributed to its upregulation. Wan et al. [21] demonstrated that ANRIL, is transcriptionally up-regulated by the transcription factor E2F1 in an ATM-dependent manner following DNA damage. In this study, we proposed a link between hypoxia and ANRIL, which are two well-known mediators of malignancy.

In this study, we investigated the expression pattern of ANRIL in osteosarcoma cells under normoxic and hypoxic conditions. Hypoxia increased the transcriptional activity and expression level of ANRIL in osteosarcoma cells. We then explored the underlying molecular mechanism that contributed to the upregulation of ANRIL under hypoxic conditions. We revealed that HIF-1α directly binds to the HREs in the ANRIL promoter region and induced ANRIL expression. HIF-1α knockdown and inhibition blunted the hypoxia-dependent transcriptional activation. HIF-1α silencing abrogated hypoxia-induced invasive capacity in osteosarcoma cells.

Apart from ANRIL, which is induced by hypoxia, previous reports have also characterized several other lncRNAs as hypoxia-responsive lncRNAs, such as lincRNA-p21 [8], LET [15], NEAT1 [22] and linc-ROR [23], which can be regulated by hypoxia and are involved in hypoxia-induced signaling transduction in cancer. These studies, in addition to the present study, suggest that lncRNAs may also play a role in hypoxia-induced signaling.

Hypoxia readily occurs in most solid tumors, and HIF-1α is upregulated in most human cancers, including osteosarcoma [10–12]. HIF-1α upregulation is associated with tumor metastases and dismal prognosis [12–14]. HIF-1α facilitated tumorigenesis by activating target genes that are involved in a wide array of cellular processes [12]. Thus, our study expanded the category of the downstream effectors of HIF-1α.

We revealed that ANRIL is a HIF-1α-inducible lncRNA and is involved in hypoxia-induced aggressive phenotype in osteosarcoma. It suggests that the HIF-1α—ANRIL pathway may be a potential therapeutic target for osteosarcoma.

## Abbreviations

lncRNA: long noncoding RNA
OS: osteosarcoma
CHIP: chromatin immunoprecipitation assay
EMSA: electrophoretic mobility shift assay
HRE: hypoxia response element
EFS: event-free survival rate
VEGFA: vascular endothelial growth factor A
ANGPTL4: angiopoietin-like 4
PGK1: phosphoglycerate kinase 1
HK2: hexose kinase 2
CAIX: carbonic anhydrase IX
